# Social Capital and Digital Divide: Implications for Mobile Health Policy in Developing Countries

**DOI:** 10.1155/2021/6651786

**Published:** 2021-01-26

**Authors:** Teng Wang, Xitong Guo, Tianshi Wu

**Affiliations:** eHealth Research Institute, School of Management, Harbin Institute of Technology, Harbin, China

## Abstract

Digital divide has been a major obstacle for mobile health services for the elderly in developing countries; to assess the potential solution to narrow digital divide among the elderly, we use data from the China Health and Retirement Longitudinal Study (CHARLS) and test for a causal role of social capital in digital access among elderly individuals in China. To handle endogenous problems associated with social capital, we introduce instrumental variable (IV) estimates in our models. Our data analysis shows that social capital facilitates increased digital access. We distinguish between two digital access patterns, an infrastructure pattern and a personal device pattern, and find that the causal effect of social capital is determined by the personal device pattern. Therefore, since family members and relatives increase digital access among elderly people, we propose a family-centered mobile health policy in developing countries.

## 1. Introduction

Noncommunicable diseases (NCDs) are the leading cause of death globally, but as the treatment and prevention of NCDs are worse in developing countries because resources are insufficient, elderly individuals there face a higher risk [1]. The characteristics of chronic diseases call for long-term and persistent self-management intervention, so patients with chronic disease need to alter their lifestyles. However, due to the fragmented health systems and insufficient funds in developing countries, the prevention and treatment for NCDs are facing more challenges [1, 2].

Mobile health (m-health) offers a potential solution to increase the efficiency of NCD treatment and prevention. Technologies such as apps and wearable devices empower patients self-tracking and self-care, specifically following and receiving instant feedback on their health, movement, and diet, improving health outcomes, and they are becoming increasingly available [3, 4]. Recent empirical research into m-health reveals that feedback, incentive, and social support mechanisms in m-health devices have helped improve health outcomes and self-efficacy among hypertension and diabetes patients [5–7]. Although mobile health is made possible by widespread mobile technology, younger, more educated, wealthier, and healthier people have an advantage in digital access to m-health; specifically, the affordability, independent usage, and ease of use have been considered as obstacles for elderly users [8, 9]. This digital divide has therefore become a main concern in m-health policy [10, 11], and it is prevalent in the developing world. For instance, in less developed countries, about 89% of urban households but only 63% of rural ones have a mobile phone [12]. One out of five people are online in less developed countries, compared with four out of five in developed countries [13].

We therefore estimate the role of social capital in the digital divide among elderly people in China. We focus on this topic for two reasons: First, although there is a proven positive relationship between social capital and health [14–18], the association between social capital and digital divide is unexamined. More importantly, increasing age means an increasing probability of chronic disease. Due to the incomplete social security system in developing countries, elderly people with chronic diseases generally face greater inequality, but among those countries with a tradition of collectivism, social capital is expected to increase digital access by providing resources for the elderly [19, 20]. Second, quantitative research on m-health policy in developing countries is lacking. ICT researchers have conducted small-sample m-health experiments to examine the feasibility of using ICT for chronic diseases. However, as m-health is a new healthcare service pattern, insufficient attention has been paid to its policy feasibility. Specifically, there is no known path of diffusion for m-health technology among underprivileged populations in developing regions [21]. The population of China is aging rapidly and seeing more NCDs: NCDs caused nearly 80% of deaths among people aged 60 or older in 2012, and in 2013 over 100 million people had at least one chronic NCD [22, 23]. Analysis of data from China will have implications for other developing countries undergoing aging and the transition of disease.

Additionally, previous studies suggested that the effect of social capital on dependent variables poses endogeneity problems, such as the mutually reinforcing relationship between social capital and local public goods [15, 24] and the relationship between living preference and wealth [25]. We measure social capital by reciprocal behavior, which is influenced by personal characteristics like altruism tendency and sympathy, latent variables that cannot be observed or controlled. To avoid the bias of coefficients on social capital and investigate the causal relationship, we use an instrumental variable (IV) approach to test and handle endogeneity problems, introducing two IVs, *Migration* and *Siblings*.

In our main results, we first find that social capital, as measured by mutual reciprocity within strong ties (relatives and friends), does have a causal effect on digital access among elderly people in China. We find two digital access patterns: the infrastructure pattern and the personal device pattern. In the infrastructure pattern, the causal effect of social capital cannot be determined since infrastructure is more sensitive to socioeconomic status (SES) indicators, while in the personal device pattern, the causal role of social capital is valid and significant in increasing digital access. Second, SES is significantly negatively associated with digital access in both patterns, a result consistent with previous studies. Age and chronic diseases are negatively associated with digital access and play a similar role to that of SES in the digital divide. This result implies that age and chronic diseases should be considered structural variables in the digital divide, and m-health in developing countries may face more difficulties than expected. Lastly, based on our findings, we propose a family-centered m-health service system in developing countries. As our results suggest that social capital has a causal effect on personal equipment, family and community can play a critical role in m-health policy to narrow the digital divide for the elderly.

## 2. Social Capital and Digital Divide

Digital divide refers to the gulf in information and communication technology access (e.g., haves or have-nots), capability (e.g., computer skills or ability to find information online), and outcomes (e.g., productivity of IT investment and use) across a variety of demographic, ethnic, geographic, and socioeconomic dimensions [26, 27]. As a measure of social structure, SES is frequently associated with the digital divide. For some researchers, the digital divide is more than digital haves or have-nots: it is part of the world of structural inequalities [28]. For example, Internet use among the middle-aged and elderly is strongly associated with SES in China, and community resources are also associated with the digital divide [10]. In the US, income, education, age, and family structure are important social determinants of online access, and older respondents were found to have lower Internet access than average [29]. However, since studies on the association between social capital and digital divide are rare and since social capital is a broad notion, we first define social capital from the perspective of private goods. Then we review the literature of social relations and digital access.

### 2.1. Social Capital: Private Goods or Public Goods?

The notion of social capital generally includes both social networks and resources embedded in those networks [30]. However, scholars do not agree on how to explain the mechanism and define the function of social capital [31]. Some researchers find that social capital motivates the community self-governance and the pursuit of collective goals by improving cohesiveness at the organization or community level [15, 24, 31, 32]. Studies following this tradition evaluate the effect of social capital on health or health resources. For instance, [17] suggests that social capital affects individual health by influencing access to services and amenities. Similarly, social capital (as measured by kindness and greeting) and social cohesion in a community increase general health [14].

Other studies in developing countries emphasize that social capital as private goods can play a more direct and significant role. In this view, resources from external ties such as relatives and acquaintances play a more critical role than collective action, and individuals rather than communities benefit; in this way, social capital is similar to individual investment [31, 33]. For instance, [20] finds that while social capital measured by organizational membership is unassociated with health outcomes in rural China, support from friends and relatives may contribute more to public goods provision. Using the number of friends as the proxy of social capital, [34] concludes that the more friends, the better one's physical and mental health outcomes. Here, we follow the private goods view in which social capital refers to actual and potential resources embedded in an individual's or social units' social networks [35, 36]. The private goods view suggests that social capital includes social networks and embedded resources. We focus on social networks rather than resources for one important reason: social networks are embedded into culture context, and collectivism is a deeply rooted cultural characteristic in developing countries, shaping individual behavior [19, 37].

### 2.2. Social Capital and Digital Access

Since studies of the association between social capital and digital divide are rare, we review work emphasizing the effect of social networks on digital access. From the private goods perspective, social networks provide resources (e.g., information and influence) that can facilitate digital access. For example, [38] finds a positive relationship between Internet use and peer effect: individuals in the proximity of others who go online will be influenced to go online themselves. Theoretically, interpersonal interactions could affect technology adoption through social learning, pressure, influence, or support (such as information). A field study in India [39] finds that farmers obtained information from and were influenced by other villagers of advice networks, and advice networks were found to increase the usage of farming information system. In another field experiment lasting for seven years in India, mothers' social networks (both strong and weak ties) were found to affect their use of ICT intervention and further reduce infant mortality [40]. In the literature of health information searching, [41] finds that teen Internet users can be health information seekers for families with low education, suggesting that young members of family may act as a potential source of digital access. Researchers aiming to increase digital access among people with low SES have found that social networks do influence underprivileged populations in developing nations, and they have also been found to increase digital access, even in less developed areas. Therefore, there is a reason to believe that social capital, via social networks, could help narrow the digital divide.

## 3. Data and Measurement

We use two databases to test the causal effect of social capital on digital access: the China Health and Retirement Longitudinal Study (CHARLS 2011) (this data is available at http://charls.pku.edu.cn/pages/data/2011-charls-wave1/zh-cn.html) and the Statistical Yearbook of China's Regional Economy (2012) (this data are available at http://www.stats.gov.cn/tjsj/tjcbw/201303/t20130318_451532.html). CHARLS is a survey of the middle-aged and elderly in China, based on a sample of households with members aged 45 or older, covering 150 countries/districts and 450 villages/urban communities, and interviewing 17,708 individuals in 10,257 households; our analysis contains 16,316 samples, and 1,392 samples were deleted due to missing variables. This data shows that, of individuals over 60, only 9.74% have Internet access and 63.92% have mobile phone access. Of individuals 45 to 59, only 20.62% have Internet access and 87.86% have mobile phone access. This low adoption rate can be considered a proxy of m-health adoption among the elderly in China today. Digital access could also act as the foundation to predict m-health access in the future because m-health services share similar ICT infrastructure for service providers and similar usage habits for users.

### 3.1. Social Capital

The private good perspective emphasizes the use of accessible resources from external networks to measure social capital in developing countries. We construct a composite score based on whether the respondent has received any help (monetary or nonmonetary) from or provided any help to others (coresident parents/parents-in-law/children/grandchildren/relatives/nonrelatives). This method is suggested and applied in previous work using CHARLS to measure social capital [42].  Figure 1 reports the distribution of social capital by SES.

### 3.2. Digital Access

Digital access can be measured by home computer ownership at the individual level, IT investment at the organizational level, and national IT expenditure at the country level [27]. Since smartphones are the current platform for m-health services, we use Internet and mobile phone access to measure digital access at the individual level. For Internet access, we ask, “Does your household have broadband Internet connection?” The majority (84%) of respondents do not. Mobile phone access is measured using the following question: “Do members of your household own the following assets?” We find that 21% of respondents have no mobile phone access at the household level. Distribution of Internet and mobile phone access by SES appears in Figures 2 and 3.

### 3.3. Control Variables

#### 3.3.1. Socioeconomic Status (SES)

Prior studies measured multiple dimensions of SES: education, occupation, access to goods and services, and household welfare. Because a single proxy could lead to unstable results [43], we use education, wealth, and residence to measure respondents' SES (see Table 1). Education is categorized into four groups (illiterate, primary, medium, and high levels). Since farmers in developing countries have no regular salary and make up a large proportion of respondents (78% have rural hukou and only 22% have urban hukou), it is difficult to accurately measure respondents' income. Expenditure is a better way to gauge income when a person's income is irregular [10, 44]. We therefore used per capita expenditure, which has also been used in other studies with CHARLS (2011). Given the urban/rural structural disparity in developing countries, we use type of hukou (urban or rural) to categorize residence.

#### 3.3.2. Chronic Diseases

The CHARLS (2011) contains 14 questions to assess chronic diseases. Comorbidity has been widely observed among chronic disease patients [45]; for instance, one-half of Chinese people aged 70 or older and one-half to two-thirds of Spanish adults older than 65 have two or more chronic conditions [1]. As suggested in previous studies [11], we note three or more cooccurring chronic diseases as an indicator of the severity of chronic disease.

#### 3.3.3. Demographic Variables

These include marriage status, sex, and age, which is subdivided into three groups (45–59, 60–74, and 75+).

#### 3.3.4. Living Arrangements

Household size and coresidence with children and grandchildren can influence digital access, since younger people are more inclined to purchase digital devices. Household size is measured by the number of people living in the same household, with a member being anyone who lived in the household for over six months in the past year. We also track whether respondents live with their adult children or with grandchildren over 16.

#### 3.3.5. Public Goods

To control for variables that may affect digital access at community and city level, we introduce public goods as control variables. Public goods related to digital access involve power supply, mobile phone base stations, etc., and we divide them into two levels, community and city. To assess public goods at the community level we follow [42, 46] and make a composite measure by asking respondents, “Does your village/community have the following type of facilities?” Fourteen facility types are listed, including basketball court, swimming pool, and outside exercise facilities. At the city level, we measure public goods by public service budget of local government (100 million yuan/10,000 people), including education, social safety net, and employment efforts. We obtain general budget and population data from the Statistical Yearbook of China's Regional Economy (2012).

## 4. Empirical Strategy

First, we use probit regression to estimate the effect of social capital. Access to Internet and mobile phone is used to estimate digital access using the following equation:

(1) $$\begin{array}{c} \text{DigitalAccess}=\beta_{0}+\beta_{1}\text{SES}+\beta_{2}\text{ChronicDisease}+\beta_{3}\text{SocialCapital}+\beta_{4}\text{Control}+\varepsilon . \end{array}$$

The variable SES is socioeconomic status including *wealth* (measured by per capita expenditure), education, and residence (measured by hukou type). *ChronicDisease* equals 1 if the respondent has three or more chronic diseases. We control for demographic characteristics, living arrangements, and public goods, denoted by *Control*. Additionally, to assess the endogeneity of social capital, we use the Wald test of exogeneity in IV-probit regression [47].

Second, given the potential endogeneity of social capital, Maximum Likelihood Estimate (MLE) will not be consistent [48], so we introduce two-step sequential estimation in models with instruments. *Migration* denotes whether the respondent left his/her birthplace and *Siblings* represents number of siblings. Our two-step IV-probit equation is specified as follows:

(2) $$\begin{array}{c} \text{SocialCapital}=\alpha_{0}+\alpha_{1}\text{Migration}+\alpha_{2}\text{Sibilings}+\alpha_{3}\text{SES}+\alpha_{4}\text{Control}+\varepsilon , \end{array}$$

(3) $$\begin{array}{c} \text{DigitalAccess}=\beta_{0}+\beta_{1}\text{SES}+\beta_{2}\text{ChronicDisease}+\beta_{3}\text{Social Capital}+\beta_{4}\text{Control}+\varepsilon . \end{array}$$

### 4.1. Instrumental Variables

Since we require a variable that associates with social capital but without a direct effect on digital access, we use *Migration* (stayers or movers) and *Siblings* as instrumental variables (IVs).

#### 4.1.1. Migration

As suggested in recent research [15, 49], *Migration* can be a proxy to measure the causal effect of social capital since it has no direct effect on infrastructure like healthcare resources. If a respondent moves away from his birthplace, the respondent is defined as a mover, otherwise as a stayer. Low population mobility, as is the case overall in China, increases the importance of interpersonal relationships and personal networks with relatives [50]. These social networks in urban communities often involve neighbors who are also work colleagues, as employees of Chinese state-owned businesses could get free housing [51]. In rural communities, people often live with extended family and their neighbors may also be relatives. Since individuals in China access resources from the social network of their place of birth, as is common in countries that are not yet totally industrialized or urbanized, stayers who remain in their birthplace can obtain more resources from existing social networks, while movers must build new social networks.

To identify movers and stayers, we ask whether the respondent's first hukou (usually obtained as an infant or child) is identical to his/her current hukou. If the respondent chooses “same as birthplace,” *Migration* equals 0 and the respondent will be marked as a migrant. According to Chinese policies, migrants need to update their hukou registration information or they may encounter some obstacles in work, education, etc. This is due to differences in social welfare policies between cites, and some welfare policies are only available for people holding local hukou; therefore, hukou can be a reliable variable to measure migration.

#### 4.1.2. Number of Siblings

Since social networks and resources are the two components of social capital, a bigger social network should have more resources for an individual. In Chinese culture, the sibling relationship is a strong tie; it involves more obligation and trust than do weaker ties between siblings in western culture [35]. We therefore use number of siblings as a proxy for strong-tie social network size; more siblings indicate a larger social network providing more social capital. For instance, information and influence obtained through social contacts help job-seekers secure higher-paying work [52, 53]. The number of siblings is measured by asking, “How many of your siblings are still alive?” As shown in Table 1, about 48.7% of respondents moved from their birthplace (movers), and respondents have an average of 3.14 *Siblings*.

### 4.2. Strength of IVs

Weak instruments can produce biased IV estimators and fail to solve the endogeneity of social capital. We address this issue by checking the results of the first-stage linear regression. A common rule of thumb considers an instrument strong if the F-statistic in the first stage is over 10 and the coefficients of IVs match theoretical assumption [54]. As shown in Table 2, the F-statistic for *Migration* and *Siblings* is 34.57 (*p* < 0.01) for social capital in both models. Additionally, the coefficients for *Migration* and *Siblings* are -0.051 (*t* = −3.01, *p* < 0.01) and 0.037 (*t* = 8.18, *p* < 0.01), respectively, indicating that *Migration* decreases resources the respondent could obtain through his/her social networks and that *Siblings* is positively associated with social capital. This result is consistent with the assumption that more strong ties result in more social capital. Taken together, we argue that *Migration* and *Siblings* are not weak IVs.

## 5. Results

### 5.1. Social Capital and Digital Divide

As shown in Table 3, the coefficient of social capital in model 1 is not significant. When the IVs are introduced in model 2, the association between social capital and Internet access is significant at 99% confidence level. The difference between these models reveals the possible bias caused by latent variables. In models with IVs, social capital is positively associated with digital access. To be specific, resources obtained from social networks increase digital access. The coefficients in models 2 and 4 are 0.79 (*t* = 3.72, *p* < 0.01) and 1.29 (*t* = 5.88, *p* < 0.01), respectively.

We turn to the Wald test of exogeneity provided in Table 3 to test if social capital is endogenous. In models 3 and 6, the chi-square equals 18.41 (*p* < 0.01) and 53.33 (*p* < 0.01), respectively, and the estimated coefficients of athrho are -0.79 (*t* = −4.29, *p* < 0.01) and −1.06 (*t* = −7.30, *p* < 0.01), respectively, indicating a negative relationship between independent variables and unmeasured variables. Hence, we reject the null hypothesis that social capital is exogenous in the 99% confidence intervals and social capital in Internet access and mobile phone access is endogenous. Compared with probit estimates for social capital in model 1 (see Table 3), the two-step IV-probit estimate for social capital is significant in model 2, suggesting that probit estimates ignore the endogenous effect of unobserved latent variables and underestimate the true effect of social capital on digital access. Taken together, we conclude that social capital is an endogenous variable.

To investigate how social capital increases the digital divide, our models in Table 3 include living arrangements. Since our measure of social capital is based on reciprocity within strong ties, household size and living situation (with adult children/grandchildren or not) may directly influence the digital access of elderly people. In the Internet model and mobile phone model, results indicate that household size and living with children/grandchildren can help increase digital access. In model 2, the coefficients of living with children (0.74, *t* = 13.46, *p* < 0.01) are relatively larger than those of living with grandchildren (0.17, *t* = 2.15, *p* < 0.05) and household size (0.06,*t* = 4.91, *p* < 0.01). Similarly, in model 5, the coefficients are 0.58 (*t* = 10.10, *p* < 0.01) vs 0.28(*t* = 3.27, *p* < 0.01) and 0.14 (*t* = 6.72, *p* < 0.01); the variance of coefficients implies that living with children can provide more digital access than living with grandchildren and the size of household. We conclude that living with offspring is an important channel by which elderly people benefit from social capital. Altogether, we conclude that social capital has a significant effect on older individuals' digital access, and support from strong ties is a path by which social capital may increase digital access.

### 5.2. SES and Digital Divide

In models 2 and 5 (see Table 3), variables of SES are strongly associated with digital access. Specifically, Internet and mobile phone access are associated with wealth and education. In model 2, a higher education level predicts higher Internet access, with coefficients of primary, medium, and high educational levels being 0.19 (*t* = 4.13, *p* < 0.01), 0.46 (*t* = 9.25, *p* < 0.01), and 0.88 (*t* = 7.67, *p* < 0.01), respectively. In model 5, they are 0.31 (*t* = 7.38, *p* < 0.01), 0.51 (*t* = 10.19, *p* < 0.01), and 0.24 (*t* = 1.73, *p* < 0.01), respectively. Another significant variable to measure SES in developing countries is urban residence, which is positively associated with digital access in both models estimated by IVs. Conversely, lack of infrastructure and of stable income can result in low access to ICT in rural areas.

We note that, in models 2 and 5, chronic diseases have a significant, negative correlation with digital access (−0.22, *t* = −4.97, *p* < 0.01 vs−0.11, *t* = −2.50, *p* < 0.05). Since healthcare costs for chronic disease patients are higher than for other elderly patients, chronic diseases can decrease the money that the individual can spend on ICT. In addition, both Internet and mobile phone access are negatively associated with age, with older people being more disadvantaged than younger people. Empirical results suggest that chronic diseases and age contribute to the structural inequality surrounding digital access for the elderly. In sum, digital access among the elderly is negatively associated with SES, which is consistent with prior studies [10, 11], and digital access is more than the difference between haves and have-nots; it also represents structural inequality. More importantly, age and chronic diseases broaden the digital divide, potentially preventing the elderly from benefiting from m-health services.

### 5.3. Robustness Checks: Instrument Validity

To satisfy the exclusion-restriction condition, *Migration* and *Siblings* are expected to be associated with social capital but to drive changes in digital access. To prove that IVs are exogenous, we perform a battery of tests. Since we have two instruments (*Migration* and *Siblings*) and one instrumented (Social capital), the estimation of an overidentified model can be performed, we introduce Generalized Method of Moments (GMM) to compare estimators and variance estimates for overidentified models (see Table 4). The results of Hansen's test are shown in Table 4. In model 7, because Hansen's *J* chi2 equals 8.04 (*p* < 0.01), we reject the null hypothesis and conclude that the overidentifying restriction (specifically, at least one of the instruments) is not valid. Model 8 supports the null hypothesis (*p* > 0.01) and we conclude that IVs are more valid in model 8 than in model 7. Therefore, the causal effect of social capital cannot be guaranteed in the Internet access model as it can in the mobile phone access model.

The difference could be partly explained by the fact that Internet access depends more on massive infrastructure investment at the community and family level than mobile phone access, which depends on an individual's capability to purchase and use personal digital equipment. As shown in Figures 2 and 3, two SES patterns influence digital access. Internet access indicates the infrastructure pattern, which is more sensitive to SES indicators than the personal device pattern represented by mobile phone access. The pattern can be further revealed by comparing the coefficients of social capital and SES in models 2 and 5. For instance, in model 5 predicting mobile phone access, demographic characteristics such as age of 60–74 and age of 75 and above have greater coefficients than the residence representing SES (−0.41, *t* = −10.54, *p* < 0.01 and −0.99, *t* = −15.76, *p* < 0.01 vs. 0.26, *t* = 4.20, *p* < 0.01), while it is the opposite in model 2 (−0.27, *t* = −0.27, *p* < 0.01 and −0.38, *t* = −5.18, *p* < 0.01 vs. 0.79, *t* = 14.07, *p* < 0.01). Considering the disparity in development between urban areas and rural areas in China, residents with high SES enjoy an advantage in access to ICT in the infrastructure pattern. Therefore, social influence (e.g., social capital) is expected to work in personal device pattern in developing countries.

## 6. Conclusion and Discussion

### 6.1. Empirical Conclusion

Our study makes several contributions. First, we determined the causal role of social capital in facilitating increased digital access, but we did not determine a causal effect of social capital on infrastructure patterns; to put it another way, our findings uncover the boundary of the social influence on digital divide. In line with prior studies, we find association between SES and digital divide among the elderly. However, age and chronic diseases also contribute to the divide, which poses a challenge to m-health policymakers in developing countries. Second, our measure of social capital is built on strong ties (relatives and friends rather than community members), and the causal relationship between social capital and digital access implies that social capital as private goods plays a critical role in China. Third, our results have implications for m-health policy in developing regions. For the elderly in developing world, despite the underprivileged are confronted with the risk of m-health divide, potential resources associated with social capital can help increase digital access. These findings remind policy makers of the importance of unique characteristics of elderly users, and the increase of access to m-health should be a priority due to the potential m-health divide.

To sum up, the main idea suggested by our study is that mobile health is more than adoption of ICT for the elderly; it is also an issue of digital equality. While prior research in the medical and IS fields focuses on urban areas and patients with relatively high SES, the underprivileged in developing countries deserve more attention. Since social capital has a positive effect on digital access, we propose that m-health policy in developing countries should fully exploit local resources including strong ties and community connections.

### 6.2. M-Health Policy Discussion

The digital divide is part of structural disparity, and continuing disparity will decrease m-health access and potentially cause an m-health divide. To avoid potential m-health divide, we suggest a family-centered m-health policy. First, family-centered m-health policy should take digital access for the elderly as a priority. Government or NGOs could provide subsidies to family members living with the elderly to increase m-health technology access. As our results suggested, social network resources should be considered to help bury structural barriers such as the urban-rural disparity and low education among the elderly. Such a family-centered m-health policy would be expected to work in developing countries. Second, family-centered m-health policy should view family as basic unit to receive m-health services to improve health outcomes. As suggested by prior research [21], m-health service implementation depends on both external and internal resources including communities and families; given the disadvantaged digital access and digital capability among the elderly, family members in developing countries are expected to facilitate the implementation of m-health services; for instance, family members could facilitate the management of chronic diseases with the guidance of general physicians.

Our findings will benefit healthcare reforms on supply side in developing countries. Due to the rapid aging and increasing threat of chronic diseases, programs like Health China 2020 in China, Family Medicine Program in Turkey [55], and Family Health Program in Brazil [56] emphasize the role of general physicians in community hospitals, but it is still unknown how to combine mobile technology and primary service. Particularly, chronic disease management requires a different service pattern compared to infectious disease services [57]; policies should pay more attention to m-health in the future for the ICT empowerment role for elderly patients.

## Figures and Tables

**Figure 1:** Distribution of social capital by residence, education, and wealth. Q25, Q50, Q75, and Q99 represent the respondents' per capita expenditure (Log) in the top 25%, top 26% to top 50%, top 50 to top 75%, and top 51% to top 99%, respectively.

**Figure 2:** Distribution of Internet access by residence, education, and wealth. Q25, Q50, Q75, and Q99 represent the respondents' per capita expenditure (Log) in the top 25%, top 26% to top 50%, top 50 to top 75%, and top 51% to top 99%, respectively.

**Figure 3:** Distribution of mobile phone access by residence, education, and wealth. Q25, Q50, Q75, and Q99 represent the respondents' per capita expenditure (Log) in the top 25%, top 26% to top 50%, top 50 to top 75%, and top 51% to top 99%, respectively.

**Table 1:** Description of variables.

	Variables	Description	Mean	Std. Dev.	Min	Max
Digital access	Dependent variables					
	Internet access	Dummy variable equals 1 if respondent's household has broadband Internet connection	0.162	0.368	0	1
	Mobile phone access	Dummy variable equals 1 if members of respondent's household own mobile phones	0.782	0.413	0	1

SES	Independent variables					
	PCE	Household members' total per capita expenditure in the past year is used as the measurement of income	2710.375	6906.97	0	233000
	Education	Education is categorized into four groups: illiterate, primary (home school or elementary school), middle (middle school, high school, or vocational school), and high (college and above)				
	IlliterateEDU	Percentage of respondents without formal education	27.29	0.819	0	1
	PrimaryEDU	Percentage of respondents who completed elementary school	39.304	0.819	0	1
	MediumEDU	Percentage of respondents who completed middle school	31.025	0.819	0	1
	HighEDU	Percentage of respondents with higher education	2.378	0.819	0	1
	Residence	Type of hukou: urban hukou is 1 and rural hukou is 0	0.22	0.414	0	1

Chronic disease	Chronic disease	Diagnosed with three or more chronic diseases (yes = 1, no = 0)	0. 186	0.389	0	1

Social capital	Social capital	Social capital is measured by a composite score. 12 dichotomous variables are measured by asking whether the respondent or spouse in the past year received/provided any economic supports from/to noncoresident parents/parents-in-law/children/grandchildren/relatives/nonrelatives. These dichotomous values are added to form a composite score	1.008	1.066	0	8

Demographic variables	Sex	Percentage of female respondents (female = 1, male = 0)	0.512	0.500	0	1
	Age	Aged 45 to 59 is middle-age level, 60 to 74 is presenior level, and 75+ is senior level				
	Aged 45–59	Percentage of respondents aged 45 to 59	55.93	0.651		
	Aged 60–74	Percentage of respondents aged 60 to 74	35.32	0.651		
	Aged above 75	Percentage of respondents aged over 75	8.75	0.651		
	Marital	Dummy variable equals 1 if married or separated and 0 if single, divorced, or widowed	0.871	0.335	0	1

Public goods	Community infrastructure	Community infrastructure is measured by a composite score. 14 dichotomous variables are measured by asking whether the community has certain infrastructure (e.g., basketball facilities), organizations (e.g., dance team), and public services (e.g., employment service center)	3.523	3.568	0	14
	Public investment	General budgetary expenditure (education, social safety net and employment effort, medical and healthcare services, agriculture forestry, and water conservation) of respondent's local government (one hundred million RMB per 10,000 people)	3.799	13.13	0.1	94

Living arrangement	HouseholdSize	Number of family members living in the same household	3.725	1.771	2	16
	Coresidence grandchildren	Percentage of respondents living with grandchildren over 16 years old	0.053	0.223	0	1
	Coresidence children	Percentage of respondents living with adult children	0.556	0.497	0	1

Instrumental variables	Migration	Equals 1 if respondent's first hukou (usually obtained as infant or child) is not his/her current hukou	0.49	0.500	0	1
	Siblings	Number of respondents' living siblings	3.140	1.929	0	11
	Observations		16316			

**Table 2:** First-stage estimates.

Social capital	Coef.	*t*-value	*p*-value	Sig
Migration	−0.05	−3.01	0.000	^*∗∗∗*^
Siblings	0.04	8.18	0.000	^*∗∗∗*^
PCE (Log)	0.05	11.04	0.000	^*∗∗∗*^
PrimaryEDU	0.04	1.98	0.050	^*∗*^
MediumEDU	0.04	1.66	0.100	
HighEDU	0.29	4.27	0.000	^*∗∗∗*^
Residence	−0.20	−8.34	0.000	^*∗∗∗*^
ChronicDisease	0.08	3.52	0.000	^*∗∗∗*^
Sex	0.04	2.36	0.020	^*∗∗*^
Aged 60–74	−0.04	−2.17	0.030	^*∗∗*^
Aged above 75	0.11	3.34	0.000	^*∗∗∗*^
HouseholdSize	−0.02	−3.97	0.000	^*∗∗∗*^
CoresidenceChildren	−0.17	−7.17	0.000	^*∗∗∗*^
CoresidenceGrandchildren	0.16	3.87	0.000	^*∗∗∗*^
Marital status	0.08	3.27	0.000	^*∗∗∗*^
Community infrastructure	0.00	1.26	0.210	
PublicInvestment(Log)	−0.07	−9.35	0.000	^*∗∗∗*^
Constant	0.67	13.51	0.000	^*∗∗∗*^
F-test	*F*(17, 16298) = 34.57] prob > *F* = 0.0000			
Observations	16316			
R-squared	0.03			

*t*-values are in parentheses.  ^*∗∗∗*^*p* < 0.01,  ^*∗∗*^*p* < 0.05,  ^*∗*^*p* < 0.1.

**Table 3:** Estimates of effect on digital access.

	Internet access			Mobile phone access		
	Probit model (1)	Two-step IV-probit model (2)	IV-probit model (3)	Probit model (4)	Two-step IV-probit model (5)	IV-probit model (6)
PCE(Log)	0.10^*∗∗∗*^	0.06^*∗∗∗*^	0.04^*∗∗∗*^	0.12^*∗∗∗*^	0.06^*∗∗∗*^	0.04^*∗∗∗*^
	(8.72)	(4.08)	(2.59)	(18.14)	(4.62)	(3.17)
PrimaryEDU	0.23^*∗∗∗*^	0.19^*∗∗∗*^	0.14^*∗∗∗*^	0.36^*∗∗∗*^	0.31^*∗∗∗*^	0.19^*∗∗∗*^
	(5.41)	(4.13)	(3.33)	(11.74)	(7.38)	(5.06)
MediumEDU	0.50^*∗∗∗*^	0.46^*∗∗∗*^	0.34^*∗∗∗*^	0.57^*∗∗∗*^	0.51^*∗∗∗*^	0.32^*∗∗∗*^
	(11.28)	(9.25)	(5.51)	(14.78)	(10.19)	(6.03)
HighEDU	1.11^*∗∗∗*^	0.88^*∗∗∗*^	0.66^*∗∗∗*^	0.61^*∗∗∗*^	0.24 ^*∗*^	0.15
	(12.99)	(7.67)	(4.28)	(5.57)	(1.73)	(1.43)
Residence	0.64^*∗∗∗*^	0.79^*∗∗∗*^	0.60^*∗∗∗*^	0.03	0.26^*∗∗∗*^	0.16^*∗∗∗*^
	(18.85)	(14.07)	(12.29)	(0.90)	(4.20)	(5.49)
ChronicDisease	−0.16^*∗∗∗*^	−0.22^*∗∗∗*^	−0.17^*∗∗∗*^	−0.02	−0.11^*∗∗∗*^	−0.07^*∗∗∗*^
	(−4.14)	(−4.97)	(−5.21)	(−0.50)	(−2.50)	(−2.65)
SocialCapital	0.02	0.79^*∗∗∗*^	0.64^*∗∗∗*^	0.10^*∗∗∗*^	1.29^*∗∗∗*^	0.81^*∗∗∗*^
	(1.52)	(3.72)	(6.50)	(7.87)	(5.88)	(17.19)
Sex	0.14^*∗∗∗*^	0.11^*∗∗∗*^	0.08^*∗∗∗*^	0.07^*∗∗∗*^	0.02	0.01
	(4.99)	(3.32)	(2.73)	(2.83)	(0.57)	(0.55)
Aged 60–74	−0.31^*∗∗∗*^	−0.27^*∗∗∗*^	−0.20^*∗∗∗*^	−0.49^*∗∗∗*^	−0.41^*∗∗∗*^	−0.26^*∗∗∗*^
	(−9.19)	(−6.68)	(−4.33)	(−17.78)	(−10.54)	(−5.77)
Aged above 75	−0.34^*∗∗∗*^	−0.38^*∗∗∗*^	−0.29^*∗∗∗*^	−0.93^*∗∗∗*^	−0.99^*∗∗∗*^	−0.61^*∗∗∗*^
	(−5.06)	(−5.18)	(−4.81)	(−20.72)	(−15.76)	(−8.50)
HouseholdSize	0.04^*∗∗∗*^	0.06^*∗∗∗*^	0.05^*∗∗∗*^	0.11^*∗∗∗*^	0.14^*∗∗∗*^	0.09^*∗∗∗*^
	(4.31)	(4.91)	(5.58)	(9.13)	(9.72)	(8.24)
CoresidenceChildren	0.62^*∗∗∗*^	0.74^*∗∗∗*^	0.56^*∗∗∗*^	0.39^*∗∗∗*^	0.58^*∗∗∗*^	0.36^*∗∗∗*^
	(15.78)	(13.46)	(10.99)	(10.42)	(10.10)	(10.28)
Coresidence grand children	0.28^*∗∗∗*^	0.17^*∗∗*^	0.12^*∗*^	0.45^*∗∗∗*^	0.28^*∗∗∗*^	0.17^*∗∗∗*^
	(4.17)	(2.15)	(1.80)	(6.96)	(3.27)	(2.67)
Marital	0.14^*∗∗∗*^	0.07	0.05	0.10^*∗∗∗*^	−0.01	−0.00
	(2.82)	(1.29)	(1.15)	(2.73)	(−0.13)	(−0.15)
CommunityInfrastructure	0.09^*∗∗∗*^	0.08^*∗∗∗*^	0.06^*∗∗∗*^	0.02^*∗∗∗*^	0.01^*∗∗∗*^	0.01^*∗∗∗*^
	(22.42)	(18.93)	(7.19)	(4.86)	(2.87)	(2.60)
PublicInvestment(Log)	0.08^*∗∗∗*^	0.14^*∗∗∗*^	0.10^*∗∗∗*^	0.05^*∗∗∗*^	0.13^*∗∗∗*^	0.08^*∗∗∗*^
	(7.54)	(7.13)	(10.79)	(4.68)	(6.40)	(9.16)
Constant	−3.22^*∗∗∗*^	−3.79^*∗∗∗*^	−2.89^*∗∗∗*^	−0.92^*∗∗∗*^	−1.82^*∗∗∗*^	−1.13^*∗∗∗*^
	(−29.71)	(−19.86)	(−12.50)	(−12.59)	(−9.66)	(−18.25)
athrho			−0.79^*∗∗∗*^			−1.06^*∗∗∗*^
			(−4.29)			(−7.30)
lnsigma			0.05^*∗∗∗*^			0.05^*∗∗∗*^
			(6.28)			(6.28)
	Wald test of exogeneity: chi^2^(1) = 18.41 prob > chi^2^ = 0.0000			Wald test of exogeneity: chi^2^(1) = 53.33 prob > chi^2^ = 0.0000				
Obs.	16316	16316	16316	16316	16316	16316
Pseudo *R*^2^	0.26	.z	.z	0.20	.z	.z

*t*-values are in parentheses. ^*∗∗∗*^*p* < 0.01, ^*∗∗*^*p* < 0.05,  ^*∗*^*p* < 0.1.

**Table 4:** Regression results GMM.

	Internet access (model 7)		Mobile phone access (model 8)	
	Coef.	t-value	Coef.	t-value
SocialCapital	0.12^*∗∗∗*^	(3.29)	0.32^*∗∗∗*^	(5.97)
PCE (Log)	0.01^*∗∗∗*^	(3.87)	0.02^*∗∗∗*^	(5.51)
PrimaryEDU	0.02 ^*∗∗*^	(2.32)	0.09^*∗∗∗*^	(8.12)
MediumEDU	0.08^*∗∗∗*^	(9.32)	0.13^*∗∗∗*^	(10.34)
HighEDU	0.29^*∗∗∗*^	(10.28)	0.05 ^*∗*^	(1.58)
Residence	0.18^*∗∗∗*^	(15.47)	0.07^*∗∗∗*^	(4.77)
ChronicDisease	−0.04^*∗∗∗*^	(−5.45)	−0.02^*∗∗*^	(−2.14)
Sex	0.02^*∗∗∗*^	(3.55)	0.00	(0.49)
Aged 60–74	−0.04^*∗∗∗*^	(−6.17)	−0.11^*∗∗∗*^	(−11.35)
Aged above 75	−0.06^*∗∗∗*^	(-5.79)	−0.31^*∗∗∗*^	(−17.73)
HouseholdSize	0.01 ^*∗∗*^	(2.53)	0.04^*∗∗∗*^	(11.43)
CoresidenceChildren	0.14^*∗∗∗*^	(13.81)	0.15^*∗∗∗*^	(10.99)
CoresidenceGrandchildren	0.02	(1.22)	0.10^*∗∗∗*^	(5.25)
Marital	0.01	(0.71)	0.00	(0.33)
Community infrastructure	0.02^*∗∗∗*^	(19.52)	0.00^*∗∗∗*^	(2.55)
Public investment (Log)	0.02^*∗∗∗*^	(7.02)	0.03^*∗∗∗*^	(6.47)
Constant	−0.26^*∗∗∗*^	(−8.11)	0.07	(1.59)
Obs.	16316		16316	
R-squared	0.11		.	
Test of overidentifying restriction:	Hansen's *J* chi2 (1) = 8.95 (*p*=0.00)		Hansen's *J* chi2 (1) = 0.62 (*p*=0.43)	

*t*-values are in parentheses. ^*∗∗∗*^*p* < 0.01, ^*∗∗*^*p* < 0.05,  ^*∗*^*p* < 0.1.

## Data Availability

The data of China Health and Retirement Longitudinal Study (CHARLS 2011) are available at http://charls.pku.edu.cn/pages/data/2011-charls-wave1/zh-cn.html. The data of the Statistical Yearbook of China's Regional Economy (2012) are available at http://www.stats.gov.cn/tjsj/tjcbw/201303/t20130318_451532.html.
